# Cost-Effectiveness of Life Cycle Cost Theory-Based Large Medical Equipment

**DOI:** 10.1155/2022/8045401

**Published:** 2022-04-16

**Authors:** Xiaoyi Chang, Yongqiang Zhao, Yuebin Li, Ting Bai, Jungang Gao, Chao Zhao

**Affiliations:** ^1^State-Owned Assets Management, The First Affiliated Hospital of Xi'an Jiaotong University, Xi'an 710061, China; ^2^School of Modern Post, Xi'an University of Posts & Telecommunications, Xi'an 710061, China; ^3^Department of Cardiology, The First Affiliated Hospital of Xi'an Jiaotong University, Xi'an 710061, China; ^4^Radiology Department (PET/CT), The First Affiliated Hospital of Xi'an Jiaotong University, Xi'an 710061, China

## Abstract

The purpose of this study is to use the life cycle cost theory to analyze the efficiency of large medical equipment in hospitals, so as to implement life cycle cost (LCC) management and solve the current problems in hospitals. The analysis model of cost benefit of large medical equipment is established, and the cost-effectiveness of 4 large medical equipment between 2019 and 2021 is investigated and analyzed. In terms of the data in each information system of hospitals, the utilization of large medical equipment is quantitatively evaluated and analyzed by life cycle theory. The results show that the Revolution 256 row has the highest revenue of 113.29%. The annual depreciation of Signa 3.0 T HDxt is the highest, amounting to 4,160,000 yuan. However, there is lack of quality control and preventive maintenance of most equipment during use. The cost and benefit of large medical equipment in hospitals are analyzed, which demonstrates that Signa 3.0 T HDxt shows better effectiveness. Too high hospital warranty cost reflects the weak maintenance strength of hospital engineering technicians. The fundamental point of the maintenance and management of large medical equipment is to strengthen the performance evaluation of medical engineering technicians.

## 1. Introduction

Large medical equipment is the reflection and significant symbol of the overall strength of contemporary hospitals. With the growing needs of management requirements, medical quality, and scientific research ability by hospitals, large medical equipment is continuously introduced and applied in the daily operation systems of hospitals to greatly promote the improvement of management, medical treatment, and scientific research levels of hospitals [1]. Besides, the in-depth use of large medical equipment in daily hospital diagnosis and treatment and the benefits it creates are the main sources of economic income of hospitals. The informatization level of hospital management becomes higher and higher with the rapid development of computer technologies in recent decades. Hospital information system (HIS) and picture archiving and communications system (PACS) are gradually promoted and applied. As a result, it is vital to accurately acquire the information about the use of existing large medical equipment in hospitals and scientifically analyze, develop, and mine the actual use, application trend, and potential of existing equipment based on existing HIS data [2]. However, medical equipment management in many hospitals is still at the stage of traditional equipment management. Manufacturers are contacted for after-sales maintenance if there are faults occurring during use. The maintenance cost is quoted by manufacturers, and whole-life insurance is purchased for large medical equipment [3]. Besides, it is expected that medical equipment has a long service life. The focus of management is on the procurement of equipment. The purchase cost of equipment is valued while the management during use is ignored. The invisible cost directly affects the operation cost of hospitals and indirectly influences the problems of the current difficulty and high cost in receiving medical diagnosis and treatment [4].

For medical equipment, the whole life process refers to the procurement, use, maintenance, and scrap of the equipment, and these links are closely related. From the perspective of hospital management system, the above-mentioned links belong to different function departments. If they are separated, for example, procurement is not considered for use; it will inevitably reduce the cost-effectiveness ratio of equipment. Full life cycle cost (LCC) includes procurement cost and maintenance cost [5]. Procurement costs can be understood as the small part of an iceberg that can be seen directly above water surface. In contrast, each cost of the maintenance cost related to LCC is like the undetectable and unrecognizable parts hidden below water surface [6]. Koneru et al. [7] reported that the consideration of only low purchase price and the ignorance of the requirements for the reliability, maintainability, safety, and environmental protection of medical equipment result in frequent medical equipment faults and even become the cause of medical negligence. After the occurrence of the faults and medical negligence, the amount of the investment needed to solve the problems is often greater [8]. The daily business data in each information system of hospitals, including the data on the benefits from patients' use of larger medical equipment, equipment usage data, and equipment operation, maintenance data, and other direct data, are combined with the auxiliary data, such as hospital human capital and energy consumption, to implement the quantitative evaluation and analysis of the utilization of large medical equipment.

Among large medical equipment, the maintenance cost of imaging equipment during use has a large proportion in lifetime expenditure. In most cases, the maintenance cost is higher than the procurement cost [9]. LCC is the basic viewpoint that guides the economic management of medical management by hospitals. The utilization of the viewpoint to comprehensively and systematically strengthen the economic management of medical equipment can create more products at less cost and then obtain good social and economic benefits [10]. The solidification of the size, parameter, performance, overall layout, and specific structure at planning and design stages generally determines the technical parameter, energy consumption level, advantages and disadvantages of the safety, reliability, and maintainability of clinical use, and maintenance cost of medical equipment [11, 12]. In order to obtain economic and reasonable life cycle cost, this study established a cost-benefit analysis model of large medical equipment and investigated and analyzed the cost-effectiveness of four large medical equipment in 2019-2021. It is hoped that the reasonable basis can be provided for medical equipment to consider the technical performance of medical equipment in the planning stage, so as to comprehensively consider the requirements of reducing maintenance costs and reducing obstacles and costs in the process of equipment remanagement.

## 2. Materials and Methods

### 2.1. Establishment of the Full Life Cycle Model

The typical research on the distribution of LCC is to divide the LCC into research and development cost, production cost, and use and guarantee cost. Of them, r&d costs only account for 10-15% of the LCC, production costs account for 30-40%, use and support costs account for 50-60%, and the proportion of other costs generally does not exceed 5% of LCC. In this study, the LCC of large-scale medical equipment is divided into purchase cost, configuration cost, use and guarantee cost, management and maintenance cost, and recovery and treatment cost. In terms of the proportion the cost of each stage, the cost of use and guarantee accounts for the largest proportion. To analyze the LCC of medical equipment, a cost estimation model is established, and then, the LCC of the system is quantitatively analyzed.

Firstly, the historical record data is statistically analyzed, and the mathematical relationship between product parameters and total cost is established according to similar principles and related principles. If the cost of the product is set as *C* and the main performance parameter set is *ϑ*, their correlation function can be expressed as follows.

(1) $$\begin{array}{c} C=f\left(\vartheta \right). \end{array}$$

Then, the equipment to be estimated is compared with the known reference equipment to find out the main similarities and differences between them. When the new equipment is similar to an existing device in function, performance, and structure, the historical cost data of existing similar equipment can be used to correct the data of the new product and finally obtain the cost of the new product to be estimated. By analog, the cost estimation equation is as follows.

(2) $$\begin{array}{c} C_{x}=C_{j}{\left(\frac{S_{x}}{S_{j}}\right)}^{\varphi }, \end{array}$$

where *C*_*j*_ is the cost of existing products similar to the new equipment, *S*_*x*_ is the performance of the new equipment, *S*_*j*_ is the performance similar to that of the new device, *φ* is the performance factor of cost, and *C*_*x*_ is the cost of the new equipment.

Medical equipment cost benefit analysis software is based on the current need for hospital cost accounting, utilizes, filter, and integrate existing considerable hospital information data to record the daily business data of large medical equipment, which lasts throughout the entire service life cycle of equipment [13]. The software plays four roles, including system administrator, device administrator, equipment maintenance personnel, and third-party system (corporate identity system (CIS) and human resource system).  Figure 1 displays the case analysis model of full life cycle.

### 2.2. Basic Information about Medical Equipment

#### 2.2.1. Large Medical Equipment Criteria

Based on *Issuance of Administrative Measures of the Allocation and Use of Large Medical Equipment*, the use of large medical equipment is improved. In addition, the utilization of complete sets of medical equipment without being included in the scope of management projects in provinces and regions but the unit price above 5 million yuan is also improved. Large medical equipment management projects are determined, adjusted, and announced by the health administrative department of the State Council jointly with other departments concerned. The projects are divided into classes A and B. The requirement for the investment, operation cost, and utilization technologies of class A large medical equipment is high, which further affects the increase in health costs. Hence, class A large medical equipment needs to be administrated directly by the health administrative department of the State Council. Besides, class B large medical equipment should be administrated by provincial health administrative departments.

#### 2.2.2. Names and Classification of Equipment

Table 1 presents the details about names and classification of various equipment.

### 2.3. Analysis of Economic Benefits

#### 2.3.1. Index Analysis Method

LCC of hospital large medical equipment refers to the procurement cost of large medical equipment purchased by hospitals and the expenditure of maintaining the equipment in normal operation before it is scrapped. The calculation method of LCC is LCC = procurement cost + maintenance cost. Procurement cost is the transaction price of the equipment purchased by hospitals, including the planning, design, manufacturing, transportation, installation, debugging, and sales profit of manufacturers at early stage. Maintenance cost refers to the fees that hospitals need to pay to ensure the normal running of the purchased equipment, including energy consumption costs, labor costs, maintenance costs, management costs, and downtime loss costs. The data used for the analysis of its cost component indexes come from state-owned asset management department, finance department, bidding and purchasing department, human resource department, HIS system, and PACS system. The cost-effectiveness of four large medical devices, Revolution 256 row, Discovery MR 750 W, Signa 3.0 T HDxt, and Optima MR 360 W, in 2019-2021 was analyzed; all the four major equipment were purchased from GE company in the United States.  Figure 2 displays the details about the sources of data information.

The depreciation cost of fixed assets is the depreciation of fixed assets drawn in accordance with regulations [14]. Based on the equilibrium allocation, the accrued depreciation amount of fixed assets is fixed into service life. The calculation method is shown in

(3) $$\begin{array}{c} A=\frac{\text{original value}}{\text{expected useful life}}, \end{array}$$

(4) $$\begin{array}{c} M=\frac{A}{12}=\left(\text{original value}\right)\times \left(\text{monthly depreciation rate}\right). \end{array}$$

In equations (3) and (4), *A* represents annual depreciation of fixed assets and *M* refers to monthly depreciation of fixed assets.

In the equipment management implemented in hospitals, equipment and commodity departments need to conduct the comprehensive calculation of equipment profits and utilization frequency combined with other relevant costs according to the corresponding utilized equipment and the charge items offered by clinical departments. In addition, the benefits after costs need to be deduced in calculating the profits produced by equipment. The calculation method is demonstrated in

(5) $$\begin{array}{c} \text{Asset utilization rate}=\left(\frac{\text{net income and expenditure}}{\text{original equipment value}}\right)\times 100\%. \end{array}$$

After the purchase of equipment, the utilization frequency index of equipment is calculated to reflect its utilization frequency and then offer the guidance on subsequent equipment procurement. In terms of the damage level of equipment, the index can reflect the damages during the utilization of equipment.

#### 2.3.2. Indicators of Benefit Analysis Method

The charging for the diagnosis and treatment by medical equipment brings benefits to hospitals, which is direct economic benefit. The evaluation of the direct benefit of medical equipment begins with the statistics and analysis of equipment revenue, equipment workload, equipment startup time, and the rate of return in equipment investment and then the comparison of the benefits of different equipment. Equipment inspection fees and treatment costs should be charged in accordance with the regulations of pricing departments. Hospitals are forbidden to formulate the charging standards independently. Therefore, the benefit analysis can be implemented by

(6) $$\begin{array}{c} \text{Annual revenue}=\left(\text{AVG medical revenue}/\text{time}\right)\times \text{times}, \end{array}$$

(7) $$\begin{array}{c} \text{Total output value of equiptment}=\text{annual output value of cycle}, \end{array}$$

(8) $$\begin{array}{c} \text{Annual revenue}=\text{business volume}\times \left(\text{cost per vist}‐\left(\text{medical revenue}/\text{time}\right)\right), \end{array}$$

(9) $$\begin{array}{c} \text{Annual profit}=\text{annual profit}-\text{annual total costs}, \end{array}$$

(10) $$\begin{array}{c} \text{Break}-\text{even business}=\frac{\text{total cost}}{\text{patient examination fee}/\text{time}}. \end{array}$$

### 2.4. Establishment of a Delay Model of Full Life Cycle

In general, random failures follow an exponential distribution, which is a special case of the Weibull distribution [15], so it can assume that the fault function belongs to an exponential distribution. Exponential distribution belongs to the form of continuous random variable distribution. The probability of Δ*t* failure in the same time period is the same, and the failure rate *γ* is constant in a time period, so the exponential distribution function is a constant failure rate function.

Thus, the failure distribution function is given as follows:

(11) $$\begin{array}{c} G\left(t\right)=1-e^{\gamma t}. \end{array}$$

The probability density function is expressed as

(12) $$\begin{array}{c} g\left(t\right)=\gamma \frac{t\gamma }{e}. \end{array}$$

The mean time to failure is calculated with

(13) $$\begin{array}{c} T=\int_{0}^{\infty }tg\left(t\right)dt=\frac{1}{\gamma }. \end{array}$$

Large-scale medical equipment has external losses and internal losses during use, and the equipment has a certain economic value in the process. At a certain stage, the residual value of the fixed assets of the equipment can be roughly estimated, which can be called the residual value of the equipment. The equation is as follows:

(14) $$\begin{array}{c} N_{a,b}\left(n\right)=\frac{{fl}^{b-h}C_{h}\left(-n\beta_{a}/e\right)\left(10-n\right)}{10}. \end{array}$$

*N*_*a*,*b*_(*n*) is the residual value function value of the equipment, and the environmental impact index is the quality of the environment in which the equipment works, which is represented by *f*. *C*_*h*_ is the purchase price of the *h*-th generation equipment, *n* is the degradation level of the equipment, and *β*_*a*_ is the degradation factor of the equipment itself.

The cost of equipment itself and workload directly affect the economic benefits of equipment. The direct benefits generated for M Hospital by large medical equipment are calculated based on the following algorithm, which is expressed by

(15) $$\begin{array}{c} \text{Return on investment}=\left(\frac{\text{In}-E_{x}}{\text{original value}}\right)\times 100\%. \end{array}$$

### 2.5. Statistical Analysis

All the data in this study are set up in Excel database and analyzed by SPSS 19.0 statistical software. The measurement data is expressed by mean standard deviation ($\bar{x}\pm s$), the counting data is expressed by the *χ*^2^ test, and the counting data is expressed by percentage (%). The difference of *P* < 0.05 was statistically significant.

## 3. Results

### 3.1. Analysis of Operation Cost

As illustrated in Figures 3–5, the 4 selected large medical equipment are compared.

Based on the above data, it is obvious that the benefit level of Revolution 256 row is the highest among that of the four large medical equipment in XX Hospital. The benefit levels of Discovery MR 750 W and Signa 3.0 T HDxt are lower than those of Revolution 256 row. The benefit level of Optima MR 360 W is the poorest with very low profit. In addition, the workload of four medical equipment and their benefits are distributed with positive correlation. With the increase of annual workloads, their benefits grow.

### 3.2. Analysis of LCC Expenditure

#### 3.2.1. Analysis of Direct Cost

Based on the equations mentioned in Materials and Methods, the actual annual depreciation fee of the equipment can be calculated. The results indicate that the annual depreciation amount of Signa 3.0 T HDxt is the highest, while that of Optima MR 360 W is the lowest, as Figure 6 shows.

Figure 7 displays the income as well as expenditure and proportion of expenditure of 4 large medical equipment in 2020.

#### 3.2.2. Analysis of Indirect Cost

After the analysis of direct cost of medical equipment, its indirect cost needs to be discussed. Indirect cost refers to various expenditures that cannot be directly included in cost category in the provision of medical health services. It needs to be allocated according to certain standards. According to the current financial regulations in hospitals, item step-by-step distribution carry-over method is adopted for department cost accounting. Hospital departments are divided into four types, including administrative logistics, medical auxiliaries, medical technology, and clinical service. The costs generated by each department at work are analyzed. Besides, various costs are apportioned by item step-by-step method according to the principles of relevance, importance, and cost benefit relationship. In this case, it is ensured that all costs are transferred to departments, which is equivalent to the deduction of the business income of clinical department. Indirect costs also include the amortization of intangible assets, for example, the software systems utilized to operate large medical equipment with huge investment and no charge. In the process of cost accounting, department allocation calculation is necessary. In addition, medical risk fund is withdrawn at 2‰ of the income of single machine business.

### 3.3. Analysis of LCC Effectiveness

Computed tomography (CT) and magnetic resonance equipment are utilized very frequently. To ensure the startup rate of the large equipment, warranty service is purchased by hospitals. Although the service is expensive, excellent maintenance service is offered in time to effectively reduce the fault rate of equipment. In terms of consumable consumption, the consumption level of CT is much higher than that of magnetic resonance. Because CT bulb tube is a high-value consumable with certain number of exposures, at least one bulb tube needs to be replaced per year according to the amount used. The average price of a bulb tube reaches as high as 1 million yuan. With good maintenance, the life of bulb tubes can be prolonged. However, bulb tubes are not covered by maintenance cost. As a result, manufacturers do not provide maintenance service for bulb tubes. According to the data in Figure 7, magnetic resonance is much less energy-saving than CT, which is related to the functions of equipment itself. According to the maintenance list offered by manufacturers, CT replacement and maintenance accessory cost amounted to 1.2 million yuan in 2019. Besides, preventive maintenance was carried out 5 times, vulnerable accessory replacement fee reached 0.5 million yuan, and man-hour cost was 1.2 million yuan. In contrast, the replacement and maintenance cost of magnetic resonance equipment accessories amounting to 1.2 million yuan in 2019 reached 0.9 million yuan with 2 preventive maintenance. Besides, the replacement cost of vulnerable accessories amounted to 0.35 million yuan and man-hour cost was 1 million yuan. The above results indicated that labor costs are generally equivalent to accessory replacement costs.  Table 2 shows a model of performance hierarchies based on the efficiency of the equipment and its performance in the process. Performance values range from 49.75 to 84.64, with the Revolution 256 row performing better in the cost-effectiveness analysis.

## 4. Discussion

Before the introduction of large medical equipment, relevant cost benefit analysis needs to be implemented to ensure the effective execution of hospital cost management. It is stipulated in the newly released medical reform policy that public hospitals must strengthen the steady development of hospitals to achieve the goal of “providing people with reassuring, high-efficient, convenient, and affordable medical health service.” In addition, the guarantee of the relationship among social responsibility, hospital development, and stable team is accelerated [16]. As a result, hospital management becomes more scientific and professional, which is the inevitable way hospitals proceed orderly and steadily. In the past, the medical equipment of hospitals is issued by the state. Hence, medical equipment may be allocated to hospitals but is restricted, which causes resource waste. Some equipment is purchased by the state with loans from the World Bank. After advanced equipment is obtained by hospitals, the lack of relevant technical personnel results in idle status and waste of the equipment. At present, hospitals can purchase medical equipment on their own. Therefore, the independent assessment of costs and benefits can be implemented before the purchase [17], which shows the significance in the strategic development of hospitals.

Hospitals need to fully take into account the financial consumption in previous purchase and subsequent maintenance, human cost, and material consumption during equipment operation. In addition, the benefits generated when the equipment is put into use also should be considered [18]. The research results show that among the four large medical devices, Revolution 256 row has the best revenue, followed by Discovery MR 750 W and Signa 3.0 T HDxt, and Optima MR 360 W has a poor revenue and low profit. The annual depreciation of Signa 3.0 T HDxt is the highest, and that of Optima MR 360 W is the lowest, which is similar to that of Sherman et al. [19]. In terms of the management of fixed assets, hospitals should firstly set up appropriate management teams or personnel to effectively manage relevant equipment. Secondly, hospitals need to establish and improve various management systems, promote responsibility-based management methods, effectively plan processes, make special files for equipment, and record its operation process. Finally, hospitals need to adopt equipment management information systems of full life cycle. The evaluation of its feasibility is conducted immediately after the purchase of equipment. In the process of equipment operation and management, real-time monitoring should be strengthened, the sharing of equipment use platform needs to be established, and reasonable arrangement for equipment use should be made. After the equipment is scrapped, a systematic evaluation should be conducted as the objective basis for future equipment purchase. Besides, the effective monitoring of single equipment needs to be strengthened to enable them to analyze cost benefits and efficiency. The data generated by the analysis offer the effective basis to the purchase and management of medical equipment [20].

Before the introduction of medical equipment by medical institutions, the corresponding positioning work needs to be carried out. Different types of medical equipment can be compared, while the performance parameters of the same type of medical equipment also can be compared [21] to provide the guidance and references for the purchase of equipment by hospitals. In some cases, some medical equipment meets the requirements only because of one of the functions. Nevertheless, other equipment possesses similar functions. Hence, a more effective analysis method needs to be adopted.

## 5. Conclusion

The following conclusions can be drawn based on the analysis of LCC effectiveness of medical equipment.

- There is lack of quality control and preventive maintenance during the use of equipment. The implementation of quality control of large medical equipment during the whole course is an effective method of the management of LCC
- The analysis of the costs and benefits of large medical equipment in hospitals demonstrates that the effectiveness of Signa 3.0 T HDxt is better
- The benefit of Revolution 256 row is the highest, reaching 113.29%. The annual depreciation amount of Signa 3.0 T HDxt is the highest, amounting to 4,160,000 yuan
- Hospital warranty cost is very high, which reflects the weak maintenance ability of hospital engineering technicians. The fundamental point of the maintenance and management of large medical equipment is to strengthen the performance evaluation of hospital engineering technicians

Based on the above conclusions, the level of cost control is directly related to the economic benefits, survival, and development of hospitals. In particular, it is important to strengthen the analysis of the cost benefits of equipment. The limitation of this study is that the corresponding horizontal comparison has not been carried out before the longitudinal comparison. From the perspective of hospitals, it is essential to establish the analysis system of the cost benefits of large medical equipment to pay less attention to procurement and more focus on management. In addition, cost behaviors need to be reasonably normalized, cost levels should be reduced, and balance needs to be increased reasonably to urge hospitals to consume less equipment as well as commodities and labor. What is more, more social benefits and economic benefits are obtained to maintain sustainable development.

## Figures and Tables

**Figure 1:** Case analysis model of full life cycle.

**Figure 2:** Details of data information sources.

**Figure 3:** Analysis of operation cost of Optima MR 360 W (1.5 T MR). (a) The annual income and expenditure of Optima MR 360 W (1.5 T MR) from 2019 to 2021. (b) The annual benefit rate of Optima MR 360 W (1.5 T MR) from 2019 to 2021.

**Figure 4:** Analysis of operation costs of Discovery MR 750 W and Signa 3.0 T HDxt (3.0 T MR). (a, c) The annual revenue and expenditure of the Discovery MR 750 W and Signa 3.0 T HDxt from 2019 to 2021. (b, d) The annual benefit rate of Discovery MR 750 W and Signa 3.0 T HDxt from 2019 to 2021.

**Figure 5:** Analysis of operation cost of Revolution 256 row (256-row CT). (a) The annual income and expenditure of Revolution 256 row (256-row CT) from 2019 to 2021. (b) The annual benefit rate of Revolution 256 row (256-row CT) from 2019 to 2021.

**Figure 6:** Annual depreciation amounts of 4 selected large medical equipment.

**Figure 7:** Proportion of expenditure of each equipment in 2020.

**Table 1:** Detailed statement of names and classification of equipment.

Classes	Company	Category	Type
Class A	GE company	1.5 T MR	Optima MR 360 W
Class A	GE company	3.0 T MR	Discovery MR 750 W
Class B	GE company	3.0 T MR	Signa 3.0 T HDxt
Class B	GE company	256-row CT	Revolution 256 row
Class A	National configuration management		
Heavy ion radiotherapy system			
Proton radiotherapy system			
PET/MR			
Cyberknife, Tomo (HD&HAD), Edge, Versa HD, and more			
Initial purchase price > $4,000,000			
Class B	Provincial configuration management		
PET/CT, contains the PET			
Endoscopic surgical instrument control system			
64-row and above CT			
1.5 T and above MR			
Linear accelerator			
*γ-*ray stereotactic radiotherapy system			
Initial purchase prices range from ￥10,000,000 to ￥30,000,000			

**Table 2:** Efficiency value and LCC value excerpts of equipment.

Type	Index	Efficiency (million)	LCC (million)
Optima MR 360 W	48	61.46	42.76
Optima MR 360 W	41	58.27	40.35
…			
Discovery MR 750 W	35	54.98	31.54
Discovery MR 750 W	28	49.75	27.65
…			
Signa 3.0 T HDxt	59	69.41	40.54
Signa 3.0 T HDxt	32	52.13	26.11
…			
Revolution 256 row	57	68.72	37.57
Revolution 256 row	64	84.64	48.39
…			

## Data Availability

The data used to support the findings of this study are included within the article.
